The article "Observation of the Effect of TTM-Based Health Information Behavior Combined with Continuous Nursing on Cognitive and Motor Function, Living Ability, and the Quality of Life of Cerebral Stroke Patients" was retracted in 2023. Reasons: unreliable results or conclusions; lack of ethics approval or compliance; concerns about the data; concerns about the peer review.

# Observation of the Effect of TTM-Based Health Information Behavior Combined with Continuous Nursing on Cognitive and Motor Function, Living Ability, and the Quality of Life of Cerebral Stroke Patients

**DOI:** 10.1155/2022/1850033

**Published:** 2022-07-01

**Authors:** Linxue Wu, Wei Jiang, Min Zhang, Guihong Fan, Guiling Li

**Affiliations:** ^1^General Medical Department, The First Affiliated Hospital of Qiqihar Medical University, Qiqihar, Heilongjiang 161041, China; ^2^Operation Room, The First Affiliated Hospital of Qiqihar Medical University, Qiqihar, Heilongjiang 161041, China; ^3^Nursing Department, The First Affiliated Hospital of Qiqihar Medical University, Qiqihar, Heilongjiang 161041, China; ^4^Nursing Institute of Qiqihar Medical University, Qiqihar, Heilongjiang 161006, China

## Abstract

**Purpose:**

To discuss the effect of the transtheoretical model (TTM) of behavior-based health information behavior combined with continuous nursing on cognitive function, motor function, living ability, and quality of life of cerebral stroke (CS) patients.

**Methods:**

540 cases of CS patients hospitalized in our hospital from June 2020 to June 2021 were selected. All the subjects were divided into the control group (270 cases) and study group (270 cases) according to the random number table. The control group was given routine nursing intervention and the study group was given TTM-based health information behavior combined with continuous nursing. The patients were paid a return visit 6 months after discharge, and their cognitive function, motor function, living ability, and quality of life were observed before and after intervention.

**Results:**

After intervention, the Montreal cognitive assessment scale score, Fugl-Meyer assessment of motor function score, Barthel index score, and short health scale score of both groups were higher than before intervention, and the study group was higher than the control group (*P* < 0.05).

**Conclusion:**

TTM-based health information behavior combined with continuous nursing has a significant positive impact on cognitive function, motor function, living ability, and quality of life of CS patients.

## 1. Introduction

Cerebral stroke (CS) is a group of diseases that causes ischemic necrosis of the brain tissue due to a variety of causes, often accompanied by severe dysfunction such as dysphagia and hemiplegia of limbs, which can lead to neurological dysfunction, cognitive decline, and motor impairment [1, 2]. The disease often occurs in middle-aged and older adults, with complicated causes and severe symptoms, which have a negative impact on patients' quality of life [3]. According to the survey, the number of patients with CS has been steadily increasing in recent years. In China, the mortality rate of CS in 2018 was 149.49/100000, about 22.3% of the total mortality rate of residents. CS has become the focus of prevention and control of cerebrovascular diseases in China [4].

The article "Observation of the Effect of TTM-Based Health Information Behavior Combined with Continuous Nursing on Cognitive and Motor Function, Living Ability, and the Quality of Life of Cerebral Stroke Patients" was retracted in 2023. Reasons: unreliable results or conclusions; lack of ethics approval or compliance; concerns about the data; concerns about the peer review.

Currently, aiming at CS patients, the nursing mode mostly focuses on nursing intervention for patients in hospital stay. After discharge, there are often problems such as unsmooth nursing connection and limited health information. Patients cannot receive adequate nursing guidance after discharge, and the prognosis is poor, which has adverse effects on patients' comprehensive rehabilitation [5]. Continuous nursing may successfully extend in-hospital nursing activities to families, continue to implement targeted nursing for patients who have not recovered from discharge, and effectively ensure that patients receive continuous healthcare services [6]. With the development of information technology, the related information sources of CS are gradually diversified. However, in the past intervention of health information behaviors, caregivers have tended to focus on patients' positive health information behaviors and may ignore the information needs that patients unconsciously put forward clearly in their daily lives, resulting in lack of relevant health information for many CS patients to guide their self-management. The transtheoretical model of behavior (TTM) is an intervention model that provides targeted behavior support in the process of behavior change through various guidance according to the needs of behavior changers [7]. TTM-based health information behavior can help patients acquire the knowledge and skills needed to establish behaviors and provide matching behavior change intervention and health information support, thus helping patients to form good self-management behaviors and correct daily bad behaviors. In this study, TTM-based health information behavior combined with continuous nursing was applied to CS patients, and targeted nursing plans were made for patients, so as to improve their quality of life.

## 2. Materials and Methods

### 2.1. Object

540 cases of CS patients hospitalized in our hospital from June 2020 to June 2021 were selected. All the subjects were divided into the control group (270 cases) and study group (270 cases) according to the random number table. Inclusion criteria were as follows: patients who meet the diagnostic criteria of CS and have the first onset of CS; stable vital signs and clear consciousness. The predicted survival was >6 months; and patients and their families knew about this study and signed written consent. Exclusion criteria were as follows: severe aphasia and hearing impairment after CS; severe organ diseases; those with poor cooperation failed to take medicine and recover as required; and those who lost follow-up or transferred to hospital halfway.

The article "Observation of the Effect of TTM-Based Health Information Behavior Combined with Continuous Nursing on Cognitive and Motor Function, Living Ability, and the Quality of Life of Cerebral Stroke Patients" was retracted in 2023. Reasons: unreliable results or conclusions; lack of ethics approval or compliance; concerns about the data; concerns about the peer review.

### 2.2. Research Methods

The control group was given routine nursing intervention: during hospitalization, followed the doctor's instructions for medication, psychological, diet, and exercise intervention were carried out, and physical symptoms were monitored. Before discharge from hospital, the importance of taking medicine on time was emphasized, and rehabilitation exercise guidance, healthy lifestyle guidance, and regular review were urged. Within 1 month after discharge, telephone follow-up was conducted once a week, and relevant guidance was given. The intervention lasted for 6 months.

The study group was given TTM-based health information behavior combined with continuous nursing: TTM teams were established, and its members included responsible nurses and rehabilitation doctors, and the questionnaire of health information behavior evaluation based on TTM was developed, as given in Table 1. After discharge, the patients were followed up by telephone once a week and visited by family once every two months until 6 months after discharge. The contents of the intervention are as follows:

1. Information collection: on the day of admission, according to the questionnaire of TTM-based health information behavior evaluation, the basic information, health information needs, health information acquisition behavior, evaluation, and utilization of health information of patients at present were known.
2. Preintention stage: 1st week of admission, the basic theoretical knowledge of CS was explained in detail; patients were encouraged to describe their inner doubts, understand their psychological problems, and successful examples were introduced. Health lectures were held, video clips were played, exercise methods were explained in easy-to-understand language, and support and encouragement were given to patients.
3. Intention stage: 2nd week of admission to planned discharge, relieve patients' doubts about rehabilitation exercise, focus on explaining the benefits of rehabilitation exercise, enhance their willingness to change behavior; and conduct lectures on psychological knowledge, explain the psychological influencing factors of behavior change, and give guidance from the psychological level.
4. Preparation stage: 2 days before discharge, the patients' mastery of the knowledge of medication, healthy lifestyle, information acquisition, and so on in the later stage of CS was known through questionnaires and interviews. In the form of distributing knowledge pamphlets, playing videos, and making action plans, medical staff explained risk factors control of CS, prevention and treatment of complications, matters for attention in home life, and functional exercise to patients in detail. Answer the questions of CS patients and demonstrate on-site rehabilitation guidance. Work with patients' families to encourage patients to make behavioral change commitments. Formulate targeted rehabilitation plans according to patients' specific conditions, for example, swallowing function training, standing balance training, gait training, and other daily life skills training.
5. Action stage: 1–3 months after discharge, answer questions of patients or their families in time after discharge and carry out telephone follow-up, door-to-door guidance, network communication, and other forms. Patients were provided with guidance on discharge rehabilitation, medication, self-care, and health information acquisition, so that patients can realize the importance of taking medicine on time, exercising scientifically and developing healthy living habits, improve patients' cognition of self-management, and correct the wrong cognition.
6. Maintenance stage: 4–6 months after discharge, through the follow-up of patients and their families, the problems in patients' self-care were found, and the detailed reasons were grasped. Adjust the rehabilitation plan for patients according to their specific rehabilitation situation and inform them of the influence of unhealthy behaviors on CS. Medical staff should monitor the patient's recovery from the disease, regularly assess the effect of the patient's behavioral changes, and inform the patient to maintain good transition.

The article "Observation of the Effect of TTM-Based Health Information Behavior Combined with Continuous Nursing on Cognitive and Motor Function, Living Ability, and the Quality of Life of Cerebral Stroke Patients" was retracted in 2023. Reasons: unreliable results or conclusions; lack of ethics approval or compliance; concerns about the data; concerns about the peer review.

### 2.3. Observation Index

The patients were paid a return visit 6 months after discharge, and their cognitive function, motor function, living ability, and quality of life were observed before and after intervention.

1. The Montreal cognitive assessment (MoCA) scale was used for cognitive function, which includes 8 areas and 11 items, including attention and concentration, executive function, memory, language, visual structure skills, abstract thinking, calculation, and orientation. A total score of 30 points, ≥26 points is normal. The higher the score, the better the cognitive function. Cronbach's *α*-coefficient of the scale was 0.813.
2. Fugl-Meyer assessment (FMA) of motor function score was used for motor function, with 33 items of upper limb function, with a total score of 66 points; and lower limb function has 17 items, with a total score of 34 points. The total score of FMA is 100 points, and the scoring method is 0–2 points. The higher the score, the better the limb motor function. Cronbach's *α*-coefficient of the scale was 0.754.
3. Barthel index (BI) was used for living ability, including bathing, eating, personal hygiene, dressing, urine control, toilet transfer, bed and chair transfer, walking on flat ground, going up and down stairs, and so on. With a total score of 100 points, the higher the score, the better the living ability. Cronbach's *α*-coefficient of the scale was 0.762.
4. The short health scale (36-item short form survey, SF-36) was used to measure the quality of life, with 36 items. 8 areas include physical function, physiological function, physical pain, general health, energy, social function, emotional function, and mental health. SF-36 has an additional area: health change. The total score of each dimension was 100 points. Calculate the average score of each dimension. The higher the score, the better the quality of life. Cronbach's *α*-coefficient of the scale was 0.850.

The article "Observation of the Effect of TTM-Based Health Information Behavior Combined with Continuous Nursing on Cognitive and Motor Function, Living Ability, and the Quality of Life of Cerebral Stroke Patients" was retracted in 2023. Reasons: unreliable results or conclusions; lack of ethics approval or compliance; concerns about the data; concerns about the peer review.

### 2.4. Statistical Methods

SPSS 22.0 software was used for analysis, measurement data were expressed as $\bar{x}\pm s$, and the *t*-test was used to analyze the comparison. Count data were expressed as a ratio, and the *χ*^2^ test was used to analyze the comparison. *P* < 0.05 was statistically significant.

## 3. Results

### 3.1. Basic Information of Patients

There was no significant difference between the two groups in terms of age, gender, education level, monthly income, and is the work or study related to medicine (*P* > 0.05) (Table 2).

### 3.2. Cognitive Function of Patients

After intervention, the MoCA scores of both groups were higher than before intervention, and the MoCA scores of the study group were higher than the control group (*P* < 0.05), as shown in Figure 1.

### 3.3. Motor Function of Patients

After intervention, the FMA scores of both groups were higher than before intervention, and the FMA scores of the study group were higher than the control group (*P* < 0.05), as shown in Figure 2.

### 3.4. Living Ability of Patients

After intervention, the BI scores of both groups were higher than before intervention, and the BI scores of the study group were higher than the control group (*P* < 0.05), as shown in Figure 3.

### 3.5. Patients' Quality of Life

After intervention, the SF-36 scores of both groups were higher than before intervention, and the SF-36 scores of the study group were higher than the control group (*P* < 0.05), as shown in Figure 4.

## 4. Discussion

With the continuous progress of medical technology, the mortality of patients with CS has decreased, but a variety of complications of patients after discharge is still inevitable. Without timely rehabilitation guidance, patients may miss the best opportunity for rehabilitation, which will seriously affect patients' cognitive function, motor function, living ability, and quality of life and eventually lead to patients cannot adapt to society [8, 9]. Therefore, CS patients still need continuous medical and health services for a period of time after discharge.

The article "Observation of the Effect of TTM-Based Health Information Behavior Combined with Continuous Nursing on Cognitive and Motor Function, Living Ability, and the Quality of Life of Cerebral Stroke Patients" was retracted in 2023. Reasons: unreliable results or conclusions; lack of ethics approval or compliance; concerns about the data; concerns about the peer review.

Continuous nursing provides health services after discharge through various follow-up methods, ensures that patients get sufficient nursing care after discharge, gives patients sufficient professional nursing guidance, and corrects patients' wrong cognition, which is continuous, reasonable, coordinated, and systematic [10, 11]. This program can help patients to establish a positive attitude, avoid complications, solve the problems encountered by patients, and help patients master home care operations, so as to make patients physically and mentally healthy [12]. In addition, most patients with CS have limited knowledge of treatment and nursing related to diseases, and they are eager to get further information and guidance related to disease rehabilitation. Health information behavior refers to the way in which individuals get information about health, health promotion activities, health risks, and diseases [13]. After discharge, patients often need to obtain a large amount of health information. Although the information itself cannot ensure the occurrence of health behaviors, health information can bring positive health behavior changes to patients [14, 15]. Therefore, in the process of nursing intervention, it is necessary to fully understand the experience of seeking health information and using health information from the perspective of patients. TTM aims to change the traditional intervention mode of behavioral events into a phased intervention mode. This theory holds that human behavior change is gradual and continuous, and it is a process consisting of 6 different stages, including information collection, preintention stage, intention stage, preparation stage, action stage, and maintenance stage [16, 17]. TTM-based health information behavior is beneficial to provide targeted behavioral support and intervention for patients, which eventually leads to behavioral change [18].

In this study, the MoCA score, FMA score, BI score, and SF-36 score of the study group are higher than those of the control group. This suggested that TTM-based health information behavior combined with continuous nursing has a significant positive impact on cognitive function, motor function, living ability, and quality of life of CS patients. Generally speaking, the routine nursing intervention mainly focuses on language and written education, lacks comprehensive assessment of patients, and neglects patients' subjective initiative, and CS patients failed to perform functional exercises in a standardized way after discharge from hospital. Continuous nursing is through the follow-up of patients and their families, patients with CS discharged from hospital are continuously monitored, and the patients and their families are instructed to master basic nursing operations as much as possible, so as to find out the problems from the patients' self-care, grasp the detailed reasons, solve the difficulties encountered in rehabilitation training, and then promote the rapid recovery of diseases [19, 20]. In the intervention of health information behavior based on TTM, medical staff understand and evaluate the basic information, health information needs, health information acquisition behavior, and evaluation and utilization of health information of CS patients through questionnaires. Medical staff provide continuous intervention nursing according to patients' state to ensure that patients' self-management ability spiraled up in different behavior stages and changed unhealthy behaviors [21, 22]. TTM-based health information and behavior combined with continuous nursing can help patients to establish effective behavior patterns, increase their motivation to change behaviors, and significantly improve their health behaviors, so as to restore their motor function and enhance their daily living ability. The combined use of the two interventions can encourage CS patients to make a commitment to behavioral change and ensure that patients can still receive timely health guidance after discharge. At the same time, after applying TTM-based health information behavior and continuous nursing to CS patients, patients' knowledge of discharged rehabilitation methods, medication precautions, method of self-care, health information acquisition forms, and other information increased, which can make patients realize the importance of taking medicine on time, exercising scientifically, and developing healthy living habits, make information support more directional, enhance patients' correct understanding of comprehensive rehabilitation, and reduce the negative impact of improper cognition on patients. This has a beneficial effect on improving the patient's quality of life.

The article "Observation of the Effect of TTM-Based Health Information Behavior Combined with Continuous Nursing on Cognitive and Motor Function, Living Ability, and the Quality of Life of Cerebral Stroke Patients" was retracted in 2023. Reasons: unreliable results or conclusions; lack of ethics approval or compliance; concerns about the data; concerns about the peer review.

## 5. Conclusion

TTM-based health information behavior combined with continuous nursing has a significant positive impact on cognitive function, motor function, living ability, and quality of life of CS patients.

## Figures and Tables

**Figure 1:** Cognitive function of patients compared with that before intervention, ^*∗*^*P* < 0.05; compared with the control group after intervention, ^#^*P* < 0.05.

**Figure 2:** Motor function of patients compared with that before intervention, ^*∗*^*P* < 0.05; compared with the control group after intervention, ^#^*P* < 0.05.

**Figure 3:** Living ability of patients compared with that before intervention, ^*∗*^*P* < 0.05; compared with the control group after intervention, ^#^*P* < 0.05.

**Figure 4:** Patients' quality of life compared with that before intervention, ^*∗*^*P* < 0.05; compared with the control group after intervention, ^#^*P* < 0.05.

**Table 1:** Questionnaire survey of health information behavior evaluation based on TTM.

TTM-based health information behavior evaluation						
Basic information						
Age	20–30 years old	30–40 years old	40–50 years old	50–60 years old	>60 years old	
Gender	Male	Female				
Education level	Below primary school	Primary school	Junior school	High school/technical secondary school	College degree or above	
Monthly income	<1000 yuan	1000–2000 yuan	2000–5000 yuan	>5000 yuan		
Is the work or study related to medicine?	Yes	No				

Health information behavior						
Health information needs						
Are you consciously and actively searching for health information?	Frequently	Occasionally	Never			
Do you know the content of health knowledge?	Yes	No				
What is your motivation to search for health knowledge? (multiple choice)	When the body is unwell	Family health reasons	When there are unclear or disputed problems in the medical process	The health promotion caught my attention	Others	
How much do you need health information?	Frequently	Occasionally	Very few	Never		
What kind of health information do you need? (multiple choice)	Diagnosis and treatment techniques and other medical information	Drug information	Nursing information	Health care information	Others	

Health information acquisition behavior						
How do you get health information? (multiple choice)	Medical institutions	Internet	Radio and television	Library	Health books, magazines and other materials	Relatives and friends
	Mobile phone SMS, WeChat	Other				
If you use the Internet to obtain health information, the ways are: (multiple choice)	Sanjiu Health Network, Health Times Network, and other health websites	Hospital website	Use search engine to search directly	Medical library website	I do not know about health websites	No internet access
Do you use online search engines (Baidu and Sina) to get health information?	Yes	No				
What do you think are the external factors that currently hinder access to health information? (multiple choice)	Less ways are provided	Information acquisition is inconvenient	Information is not provided in time	Lack of information I need	Others	
What are your own limitations in obtaining health information? (multiple choice)	I do not know where to find information	Too much information, I do not know what to use	Fear of false information	Personal economic conditions	Personal cultural quality is not high	Others
Main obstacles for you to search for health information	Busy at work, no time	Internet access is inconvenient	Insufficient information retrieval skills	Lack of computer level	Others	
Evaluation and utilization of health information						
When you obtain health information, will you consider the authority of the information?	Yes	No				
When you obtain health information, will you consider the authenticity of the information?	Yes	No				
When you obtain health information, will you consider the novelty of the information?	Yes	No				
Will the acquired health information affect your judgment on your illness?	Yes	No				
Can you fully understand the health information you have obtained?	Fully understand	Most understand	Understand a little bit	Do not understand at all		

The article "Observation of the Effect of TTM-Based Health Information Behavior Combined with Continuous Nursing on Cognitive and Motor Function, Living Ability, and the Quality of Life of Cerebral Stroke Patients" was retracted in 2023. Reasons: unreliable results or conclusions; lack of ethics approval or compliance; concerns about the data; concerns about the peer review.

**Table 2:** Basic information of patients (*n*, %).

Group	Control group	Study group	*χ* ^2^ value	*P* value
Age (years)			1.640	0.802
20–30	102 (37.78%)	98 (36.30%)		
30–40	42 (15.56%)	43 (15.93%)		
40–50	41 (15.19%)	37 (13.70%)		
50–60	35 (12.96%)	45 (16.67%)		
>60	50 (18.52%)	47 (17.41%)		

Gender			1.465	0.226
Man	90 (33.33%)	77 (28.52%)		
Woman	180 (66.67%)	193 (71.48%)		

Education level			0.855	0.931
Below primary school	21 (7.78%)	17 (6.30%)		
Primary school	15 (5.56%)	16 (5.93%)		
Junior school	55 (20.37%)	51 (18.89%)		
High school/technical secondary school	50 (18.52%)	49 (18.15%)		
College degree or above	129 (47.78%)	137 (50.74%)		

Monthly income (yuan)			0.968	0.809
<1000	68 (25.19%)	72 (26.67%)		
1000–2000	77 (28.52%)	70 (25.93%)		
2000–5000	93 (34.44%	100 (37.04%)		
>5000	32 (11.85%)	28 (10.37%)		

Is the work or study related to medicine?			2.173	0.140
Yes	143 (52.96%)	160 (59.26%)		
No	127 (47.04%)	110 (40.74%)		

## Data Availability

The data used and/or analyzed during the current study are available from the corresponding author upon request.
